The article "Information Collection, Analysis, and Monitoring System of Children's Physical Training Based on Multisensor" was retracted in 2023. Reasons: signs of a paper mill; suspected computer-generated content; unreliable results or conclusions; lack of ethics approval or compliance.

# Information Collection, Analysis, and Monitoring System of Children's Physical Training Based on Multisensor

**DOI:** 10.1155/2022/6455841

**Published:** 2022-05-12

**Authors:** Zhonglin Zhang, Jiajia Xu, Chenggen Peng, Yuping Chen

**Affiliations:** ^1^College of Sport, Huaiyin Normal University, Huaian, 223001 Jiangsu, China; ^*^2^*^ College of Pre-Primary Education, Woosuk University, Wanju-gun, 55338 North Jeolla Province, Republic of Korea; ^*^3^*^ College of Sport, Hunan Agricultural University, Changsha, 410128 Hunan, China

## Abstract

In order to obtain more children's physical training information and improve the accuracy of children's physical training monitoring, a multisensor-based children's physical training information collection, analysis, and monitoring system is proposed. In the process of physical training and sports training, people's physical training information collection is directly related to the level and effectiveness of physical training. With the combination of multisensor concept and sports training information collection, it can collect the key index data of sports mobilization in real time with the help of multiple sensors and information technology. Taking children's physical training as the object, this paper designs a multisensor physical training data information acquisition terminal, collects different training characteristic data with the help of multisensor equipment, and then comprehensively analyzes and monitors the physical information with the help of certain fusion technology, so as to construct a human posture recognition algorithm based on children's physical training information acquisition. Support vector machine and decision tree are used to classify children's different physical exercise states, and a relatively perfect algorithm architecture of human posture recognition is constructed. The results show that for two decision trees, each decision tree is trained with a total of 675 groups of data, and a total of 342 groups of data are verified and pruned. The two decision trees take 7.17 s and 7.32 s to complete the training process, respectively. It can be seen that when the number of training groups is equal, the training time of the two placement methods is close, so it can be considered that the two placement methods have little effect on the training speed of decision tree. The experimental data show that the design of children's physical training monitoring system in this paper has a certain market value.

## 1. Introduction

In the process of sports training, the collection of athletes' physical training data information is directly related to the improvement of athletes' training level. Applying the concept of multisensor to training data acquisition and information fusion technology, we can collect and sort out the key data information of athletes' physical training with the help of multisensor, camera, and other equipment [1]. Multisensor human-computer interaction system is a process system through the mutual blending, understanding, and information feedback of human, computer, and specific environment.  Figure 1 is a manufacturing method of a physical training monitoring system. There are some differences between children's physical training and ordinary athletes' training requirements. Because there is great uncertainty in the training process of children's group, it can not be carried out simply through single indicators and traditional evaluation techniques. Children's complex human and environmental factors should be fully considered [2, 3]. In the process of physical training, compared with mature athletes, children's body presents a more special physical movement state of randomness, complexity, and diversity. From the perspective of machinery and equipment, the human body is mainly a complex system composed of various subsystems. These different subsystems have their own functions and characteristics and have close contact and communication with each other. On the basis of mutual coordination and connection, they form the movement process of human body. Therefore, children's physical training behavior has complex characteristics. As an inevitable trend in the field of intelligent interactive control in the future, multisensor human-computer interaction system requires that the system based on multisensor can comprehensively analyze human action modes, characteristics, and connections. Human posture recognition system can be used as the application direction of human-computer intelligent interaction of specific pattern recognition and provide decision-making data basis for human-computer intelligent interaction control and human motion behavior pattern analysis [4].

At present, there are relatively many research topics in the field of human sports training model simulation, by constructing athletes' human training model to simulate the training data of athletes' training process, including athletes' training steps, speed, heart rate, acceleration, and other physical dynamics. By mastering these data information in real time, we can further grasp athletes' sports level, which can provide reliable data support for improving athletes' sports effect. However, the current research is more true from the external movement performance, and there is little research on the role of muscle activity and internal performance in the process of human training, so that there is relatively little data collection and fusion analysis. In the 1970s, a technology based on data acquisition and fusion appeared, which seems to be to fuse the data information collected by a variety of devices into an effective combination for a certain research institute, for example, neural network algorithm, decision tree theory, information theory, and statistical reasoning. These information fusion technologies can comprehensively analyze the data according to certain criteria and algorithms and obtain relatively accurate prediction results of the research object on this basis. Based on this, taking children's physical training as the object, this paper designs a multisensor physical training data information acquisition terminal, collects different training characteristic data with the help of multisensor equipment, and then comprehensively analyzes and monitors the physical information with the help of certain fusion technology, so as to construct a human posture recognition algorithm based on children's physical training information acquisition. Support vector machine and decision tree are used to classify children's different physical exercise states, and a relatively perfect human posture recognition algorithm architecture is constructed [5, 6].

## 2. Literature Review

Bowler and others have realized the recognition of PA (physical activity) by using five acceleration sensors and can judge the intensity of some sports. In this document, the author also compared the accuracy of learning and judgment using subject dependent training (94.6%) and subject independent training (56.3%) [7]. Hurot and others also built a wireless sensor network based on five sensors for human activity recognition, including 13 actions such as jumping, going up and down stairs, and walking left and right. After the movement lasted for 10 seconds, the recognition accuracy also reached 99.2% (SVM), and the accuracy was very ideal [8]. Park and others used the method of machine learning and fuzzy classification in the research of human action recognition based on wearable sensors, in order to find a general human action recognition model that can adapt to any individual [9]. Xiong and others used recursive PCA, LDA, and eHAR classifiers to adapt to different people by constantly changing the model. Although the accuracy of this recognition method is not high (80% ~90%), it has wide adaptability [10]. Scotti and others used multiple sensors to jointly identify human actions, which has the advantages of multiple data dimensions, more and more detailed actions, and higher robustness. At the same time, by using a specific combination of sensors, we can recognize the specific and subtle actions of the human body, such as distinguishing the upper limb posture recognition and the lower limb posture recognition, which can make the human motion recognition technology better applied in different fields. Selecting different kinds of sensors such as pressure, geomagnetic meter, and temperature can realize more recognition functions [11]. In addition, multisensor is different from single sensor to recognize human actions. One essential advantage is that multisensor recognition, based on wearable sensor network, can study the interaction between multiple people, which can not be realized by using only a single sensor.

Because the research in this direction started late and has more far-reaching social significance than identifying the actions of a single person, it has high research value. However, there are also many problems when using multiple sensors for recognition: first, for different target actions, how to use the number and position combination of sensors to effectively recognize all target actions is a problem that needs to be considered; secondly, the amount of data generated by multiple sensors will be much more than that of a single sensor, which will increase the amount of computation. How to reduce and reduce the amount of computation without losing the recognition accuracy is a test; finally, what algorithm or recognition method can better realize the real-time performance of action recognition for a large number of data is also a problem worthy of study [12]. Because the human motion recognition based on sensor can directly obtain the relevant data of motion state and can provide the basis for studying the law of human motion and the technical characteristics of sports, it is very appropriate and effective to study the human motion during sports, analyze and study it, and realize it by using sensor technology. At the same time, in the current research, there are few papers that use multisensor to distinguish and study the technical actions of basketball, so the research direction can be developed and studied [13]. Through the research of human motion recognition at this stage and the reading of previous papers, human motion pattern recognition mainly uses the classification method of machine learning to classify the collected motion data, so as to realize the recognition of human motion. According to the literature, the flow of the general method of human motion recognition using machine learning method is divided into data acquisition, data preprocessing, feature selection, feature extraction, training, recognition, and evaluation, and the flow chart of motion recognition can be sorted out (see Figure 2).

## 3. Research Methods

### 3.1. Overall System Design

The purpose of applying multisource information fusion technology to athlete training information system is to obtain various parameters of human movement process, fuse, and analyze these parameters, so as to provide effective and helpful decision-making data and technical guidance for athlete training. The system architecture is shown in Figure 3.

The system includes four layers: data layer, feature layer, feature fusion layer, and decision layer. It can be seen from the figure that the scientific training technical guidance or sports level is the result of fusion analysis based on the information acquisition and processing of athletes' human movement process. Therefore, the main research of this paper is how to obtain the multiobjective and multiparameter data in the process of athlete training for effective fusion analysis [14].

### 3.2. Acquisition and Processing of Children's Human Movement Information Data

#### 3.2.1. Acquisition of Human Motion Information Data

The information in the process of human movement itself is a complex nonlinear process parameter, which involves kinematics, dynamics, physiology (electromyography), and so on. Different models have different inertia parameters. The camera is used to obtain human kinematics parameters, and the force test platform is used to obtain external force parameters.

*(1) Kinematic Information Acquisition*. The kinematic parameters are mainly obtained by high-speed camera, three-dimensional video recording, and other technologies.

For high speed photography technology, due to different shooting methods, the measurement range of shooting is also different. When obtaining information, the shooting method depends on the athlete's training program. The plane fixed camera shooting method has a small measuring plane range and is suitable for items in the movement of the measured body on a plane, such as long jump and take-off. The plane tracking shooting method has a small measurement range and is larger than the fixed machine shooting method. Because the measured object cannot keep a uniform linear motion all the time, it is inevitable that it is different from the camera speed and obtains erroneous measurement results. It is generally suitable for sports projects with long cycle distance and large measurement range. The method of three-dimensional fixed camera shooting is mainly to shoot the motion process of the same tested body from different angles at the same time. Only two cameras can shoot at the same time. The graphics obtained from cameras from different angles at the same time are digitized, and the obtained motion parameters can be applied to sports such as shot put [15].

For 3D video technology, three-dimensional video recording technology is based on the principle of three-dimensional space reconstruction. Information collectors can shoot with more than two cameras set in a stable and unchanged position. The three-dimensional space coordinates obtained by the linear transformation algorithm make a high-precision calibration framework of at least six known coordinate points, and the camera angle difference is generally 90 degrees. The shooting method has large measurement space and simple structure. It is suitable for gymnastics, ball games, track and field, and other sports.

*(2) Dynamic Information Acquisition*. In the process of motion, dynamic information can be obtained through sensors, which has an important impact on motion analysis. Dynamic parameters generally include human body displacement, plantar pressure, joint force, angle, and acceleration, which can be obtained by force sensor, displacement sensor, speed sensor, accelerometer, inertial sensor, and goniometer. At present, the six-dimensional force test platform developed by the research institute can be divided into three modules: force sensor, signal processing module, and computer module. The measurement area is large, and the force cabinet data and three-dimensional spatial data can be obtained at the same time.

*(3) EMG Information Acquisition*. Electromyography is a pattern obtained by processing weak electrical signals released by nerves and muscles during exercise. Through the EMG measuring instrument, according to the EMG electrode, the relaxation and contraction degree of human muscle and other data are obtained. After the processed EMG analysis, the athletes can be scientifically guided, and the training level can be improved. Due to different electrode objects, EMG signals can be divided into surface EMG and needle electrode EMG. During exercise training, surface EMG detection is mostly used because this method has no damage to the human body and only measures the EMG data on the surface of human skin [16].

#### 3.2.2. Human Motion Information Data Processing

The human motion data collected by the sensor is given based on the reference system of each sensor. Since human motion cannot be described according to the reference system of the sensor, such source data cannot be used directly. Therefore, the coordinate system transformation mode is introduced, after completing the coordinate system transformation, according to the general process of human motion recognition, the source data used for human motion recognition needs feature extraction. This section will introduce the digital features used in this topic.

*(1) Data Coordinate System Transformation*. For human motion, to know the specific motion form, we must first establish a coordinate system according to the direction of human motion, which is represented by the sensor installed on the human body. According to the working principle of the sensor, the angle data returned by the sensor is Euler angle, which represents the difference between the current motion coordinate system and the ground coordinate system. Therefore, the coordinate system of all sensors can be unified as the ground reference system, as shown in Figure 4.

All sensors will have an initial angle according to the standing position and posture. The analysis principle of each sensor is the same, so any sensor is analyzed. It can be proved by calculation that the point coordinates *Ab*(*xb*, *yb*, *zb*) represented in the *O*_*b*_-*X*_*b*_*Y*_*b*_*Z*_*b*_ coordinate system are transformed into the coordinate transformation matrix of the point *Ag*(*xg*, *yg*, *zg*) under the *Og* − *XgYgZg* coordinate system. According to the coordinate transformation matrix, the coordinates can be mapped to a unified ground coordinate system. During the experiment, due to the site, the movement direction will not be consistent every time, and it is impossible for the tested personnel to move in the same direction every time. Since the ground coordinate system takes the vertical direction downward as the *z*-axis, and the personnel movement is also carried out under the influence of gravity; the two are consistent. Therefore, the travel coordinate system *O*-*XYZ* is established with the vertical direction as the *z*-axis, the personnel travel direction as the *x*-axis, and the personnel's right hand direction as the *y*-axis. Therefore, it is necessary to transform the point coordinates *As*(*xs*, *ys*, *zs*) in the sensor coordinate system *Os*-*XsYsZs* to the point *A*(*x*, *y*, *z*) under the travel coordinate system *O*-*XYZ* to recognize the action. It is noted that if the coordinate system is transformed to the ground coordinate system first and then to the travel coordinate system, it will undergo two coordinate transformations, which will increase unnecessary overhead [17, 18]. Therefore, the way of direct change is considered here. In one coordinate system O1, it is known that the direction vectors of the *X* and *Z* axes of the other coordinate system *O*2 are as follows:

(1) $$\begin{array}{c} \begin{array}{c} {\bar{n}}_{x}=\left(x_{x},y_{x},z_{x}\right),\\ {\bar{n}}_{z}=\left(x_{z},y_{z},z_{z}\right). \end{array} \end{array}$$

The attitude angle of the object in O2 coordinate system expressed in O1 can be calculated. The solution formula is shown as follows:

(2) $$\begin{array}{c} \theta^{\prime }=\left\{\begin{array}{c} \arccos\frac{\sqrt{x_{x}^{2}+y_{x}^{2}}}{\sqrt{x_{x}^{2}+y_{x}^{2}+z_{x}^{2}}}⟶z_{x}\geq 0\\ \pi ‐\arccos\frac{\sqrt{x_{x}^{2}+y_{x}^{2}}}{\sqrt{x_{x}^{2}+y_{x}^{2}+z_{x}^{2}}}⟶z_{x}<0 \end{array}\right.,\\ \psi^{\prime }=\left\{\begin{array}{c} \arccos\frac{x_{x}}{\sqrt{x_{x}^{2}+y_{x}^{2}}}⟶y_{x}\geq 0\\ \pi ‐\arccos\frac{x_{x}}{\sqrt{x_{x}^{2}+y_{x}^{2}}}⟶y_{x}<0 \end{array}\right.. \end{array}$$

For the method of determining the human motion coordinate system, firstly, take the standing human body posture as the benchmark, and the tested person first keeps standing vertically for 2S. At this time, the mean value of attitude angle can be calculated through the sensor data, and the mean value of static attitude angle and static acceleration can be calculated at the same time. Considering that it is only affected by gravity at rest, the direction of maximum acceleration is the direction of gravity acceleration. At this time, the representation of the acceleration vector in the coordinate system can be obtained according to the acceleration components in three axes, and the direction of the vector is the *z*-axis direction in the human motion reference system.

Then, make the subject lie down on the ground and keep the left and right orientation unchanged. At this time, the direction of gravity acceleration is the negative direction of *x*-axis. The vector of *x*-axis direction can be calculated according to the direction of gravity acceleration. The means to verify the measurement accuracy is to calculate the inner product of the above two coordinate axes. The method to obtain the *y*-axis vector is to use the outer product of the *z*-direction vector and the *x*-direction vector. Since the direction vector coordinates measured above are expressed in each sensor coordinate system, the sensor coordinate system can be converted into human motion coordinate system at one time. Based on the human motion coordinate system, the acceleration in the process of human motion can be expressed in the same reference system as the direction of human motion, which is the basic reference system based on this experiment [19, 20].

*(2) Signal Characteristics*. Signal feature is a quantity that can describe the characteristics of statistical variables from many different angles based on the overall data. It is divided into time-domain feature and frequency-domain feature. Each section of sampled data describing human motion contains rich time-domain and frequency-domain features. This paragraph introduces the digital features commonly used in the field of human motion recognition. The time-domain features commonly used in human motion recognition include sample mean, sample variance or standard deviation, correlation coefficient, and energy between two axes.

The sample mean is calculated as follows:

(3) $$\begin{array}{c} \mu =\frac{1}{n}\overset{n}{\underset{i=1}{\sum }}a_{i}. \end{array}$$

The sample variance is calculated as follows:

(4) $$\begin{array}{c} \sigma^{2}=\frac{1}{n}\overset{n}{\underset{i=1}{\sum }}{\left(a_{i}-\mu \right)}^{2}. \end{array}$$

Standard deviation is calculated as follows:

(5) $$\begin{array}{c} \sigma =\sqrt{\frac{1}{n}\overset{n}{\underset{i=1}{\sum }}{\left(a_{i}-\mu \right)}^{2}}. \end{array}$$

The covariance is calculated as follows:

(6) $$\begin{array}{c} \mathrm{cov}\left(\alpha ,\beta \right)=E\left[\left(\alpha -E\left(\alpha \right)\right)\left(\beta -E\left(\beta \right)\right)\right], \end{array}$$

where *E*(*a*) and *E*(*β*), respectively, represent the expectations of two different variables and the correlation coefficient is shown as follows:

(7) $$\begin{array}{c} \rho =\frac{\mathrm{cov}\left(\alpha ,\beta \right)}{\sigma_{\alpha }\sigma_{\beta }}. \end{array}$$

Frequency domain features are usually calculated by fast Fourier transform (FFT), which is used to find the characteristics of frequency and periodic information in the signal. Kurtosis indicates the sharpness of the peak shape of a section of sample value. The larger the kurtosis value, the sharper the signal shape. The smaller the kurtosis value, the flatter the shape. It is usually processed by subtracting 3 to make the waveform kurtosis of standard normal distribution 0. The calculation of kurtosis is calculated as follows:

(8) $$\begin{array}{c} \text{Kurtosis}=\frac{\left(1/\left(n-1\right)\right)\sum_{i=1}^{n}{\left(\alpha_{i}-\mu \right)}^{4}}{\sigma^{4}}-3. \end{array}$$

Skewness measures the deviation of the signal shape from the central axis of the normal signal. Skewness < 0 is the left deviation of the waveform, and Skewness > 0 is the right deviation of the waveform. Calculation formula is as follows:

(9) $$\begin{array}{c} \text{Skewness}=\frac{\left(1/n-1\right)\sum_{i=1}^{n}{\left(\alpha_{i}-\mu \right)}^{3}}{\sigma^{3}}. \end{array}$$

## 4. Result Discussion

### 4.1. Evaluation of Children's Physical Training Action Recognition Results

#### 4.1.1. Data Sampling

According to the collected data, the movement frequency of human limbs is below 10 Hz. Therefore, according to Nyquist sampling theorem, the sampling frequency above 20 Hz can effectively represent the movement state of human body. Here, the sampling frequency 50 Hz is used to collect the data of human body movement. The duration of each section of data to be processed is 5S. During the 5S period, the actions of free throw, jump shot, take-off, and standing only last for one cycle. As the action cycle of other actions is short, multiple action cycles will be completed within 5S. After the sampling is completed, the action is periodically segmented through the periodic segmentation method described in Chapter 3, and the data on each cycle is processed with digital features to take the mean value. For jumping, walking, running, standing, dribbling, and other movements, because the data needs to be collected for many times, the basket frame is not necessary, and there are more personnel mobility in the basketball court and less spare space, the data collection is carried out not only in the basketball court but also in the playground, open space, and other flat places.

Since the reference system for identifying human motion in this paper is based on human motion coordinate system, which needs experimental test, it is necessary to calibrate and calculate the initial value of human motion coordinate system. Since the *y*-axis direction points to the right direction of human movement, it is difficult to measure the accurate direction, but the *x*-axis and *z*-axis directions are easy to measure. Therefore, the *y*-axis is calculated by making the vector outer product according to the input of the *x*-axis and *z*-axis direction vectors. For *z*-axis direction measurement, before human motion data collection, draw the straight line to be moved with chalk on the ground. The measured person stands vertically facing the moving direction to be moved and keeps standing stably for 5S. Take the most stable 2S data, calculate the average value of the three-axis gravitational acceleration direction, and obtain the vector coordinates of the *z*-axis direction through the data of the three axes. For *x*-axis direction measurement, place the yoga mat parallel to the movement direction indication line drawn on the ground, and the tested person lies flat on the yoga mat parallel to the yoga mat to keep the lying down movement stable. At this time, relative to the sensor, the direction represented by the gravity direction is the opposite direction of the movement direction of the human body [21]. Through the calculation of the most stable 2S data in the 5S stable action, the vector coordinates can be obtained, and the inverse can be used to obtain the vector coordinates in the *x*-axis direction. After measuring the *x*-axis and *z*-axis directions, the verticality is judged by calculating the included angle of the vector. Due to the measurement error, it is considered that as long as the included angle of the two vectors is between 88° and 92°, it is considered to be vertical.

#### 4.1.2. Sensor Data Error Evaluation

Place the sensor naturally on the plane, collect the data measured by the sensor, calculate the mean and variance of the measured gravity acceleration for the sensor data, and calculate the mean and variance of the measured angle data. The stability of the sensor measurement data is determined through these two digital features. For each sensor, different placement angles are used to maintain the stability of the measurement environment. Through three measurements, the mean and variance of the sensor data obtained each time are investigated to determine the stability of the sensor measurement data. The measurement results are shown in Table 1.

From the digital characteristics obtained by the sensor, it can be seen that when the sensor is stationary, the data returned by the data fluctuates less, and the same sensor is placed in the same position and sampled at different times. The result is relatively stable, and there is no obvious measurement data drift. Therefore, the sensor data is within the allowable error range and can be considered accurate.

#### 4.1.3. Subjects

In the experiment, 10 normal and healthy students were selected for data collection, including 7 boys and 3 girls. Each person completed 9 movements, respectively, and each person collected 30 times of each movement. Among them, 15 groups of sensors were worn on the left foot, and 15 groups of sensor data were worn on the right foot. Each action has a total of 300 groups of action data, which are divided into two sensor wearing methods. In this study, 300 groups of data of each action obtained from the experiment are divided into training set, verification set, and recognition object data set by setting aside the experimental data. The training set data is used for the training of classification algorithm. The validation set data is used as the basis for decision tree pruning. Finally, the objects in the recognition object data set are classified and recognized. For each group of jumping action and jump shot action, it is necessary to estimate the high jump height as the input parameter of weight loss recognition. Here, the take-off height is estimated according to the visual height of both feet from the ground, with the unit of CM. The method of visual estimation is to place a vertical ruler beside the tested person to keep the line of sight level. The eyes, the scale of the ruler, and the height of the tester's heel off the ground are at the same level, and the reading is taken when the jumper reaches the highest point.

#### 4.1.4. Experimental PC Configuration

Table 2 shows the experimental PC configuration.

#### 4.1.5. Experimental Results

*(1) Timing Mode*. This chapter not only analyzes the recognition accuracy of the algorithm but also analyzes the running time of the algorithm. Here, the timing method is through the timing function, write down the start time before a step, and then start the step immediately; write down the end time immediately after you finish a step.

*(2) Weightlessness Feature Extraction Results*. Since the weightlessness feature recognition algorithm only investigates the component of trunk acceleration, it has nothing to do with the left and right sides of lower limb sensors. Here, 50% of 300 groups of data, that is, 150 groups of data, are used for training. The start limit interval obtained from training is (-1.7496, 0.2602), where *μ* = −0.7447, *σ* = 0.2792, and *σμ* = 0.1673. The end limit interval obtained by training is (-2.9523, 0.2459), where *μ* = −1.3532, *σ* = 0.4529, and *σμ* = 0.2404.

The recognition accuracy results of the remaining 150 groups of jump data after training are shown in Table 3.

Through numerical analysis of two samples with recognition errors, it is found that these two data are from girls' jump shots, with low jump height and unstable acceleration during jumping, so the weightlessness time is less than 0.285 s.

*(3) Time Result*. Due to the weightlessness feature extraction, the data need to be traversed from back to front, and only a small amount of data need to be averaged, which has high efficiency. The identification time of 150 groups of data in the verification set is counted, and the average time-consuming results are shown in Table 4.

For 150 groups of data in this subject, the average time of weight loss feature recognition in each group is 0.03327 ms.

*(4) Feature Vector Extraction Results*. The features of the original data are extracted, and the classification results are classified based on these feature vectors. The nine technical movements involved in each subject are as follows: standing, taking off, shooting, jump shot, dribbling, walking dribbling, running dribbling, walking, and running. The *z*-axis mean of trunk sensor, *z*-axis kurtosis, *z*-axis skewness, *XY*-axis cross-correlation coefficient, *yz*-axis cross-correlation coefficient and *y*-axis standard deviation of forearm sensor, *x*-axis standard deviation, *z*-axis standard deviation of leg sensor, and take-off feature are extracted, respectively.

*(5) Decision Tree Classification Results*. In this study, the data set is divided into two parts. One part is that the lower limb sensor is placed on the same side as the manipulator, and the other part is placed on the opposite side of the manipulator, taking 50% of each, that is, 75 groups of data, and two decision trees are generated, respectively. According to 25% of the data on each data set, 38 data are taken as the verification set, and the remaining 37 data are taken as the identified objects. Therefore, both decision trees include 75 training data as training samples, 38 verification sets as pruning basis, and 37 objects to be identified as the standard verification set for the final generalization ability evaluation. The accuracy on the verification set is shown in Tables 5 and 6.

Among them, “misidentification of other actions” means that other actions are misidentified as this action, and “error” means that this action is identified as other actions. The error condition is to describe the specific error type in the “error” column. The calculation method is that assuming that other actions are wrongly recognized as this action, the total number of data recognition groups is added by 1, and then, the correct recognition number is divided by the total number to obtain the recognition accuracy. It can be seen that in the recognition rate of the verification set, the recognition rate of walking, walking dribbling, and running is low. In fact, the decision tree has been pruned. For example, one of the nodes classifies the actions of two running dribbles in the training set, which are divided into running and running dribbles. Here, the pruning operation is carried out according to the recognition results of the verification set. After pruning, it also has a better recognition rate for the identified object data set. From the comparison between the two tables, it can be seen that the average recognition accuracy before pruning is 93.85% for the same side mode and 94.64% for the different side mode, respectively. The accuracy of the different side placement is slightly higher, but the difference between the recognition accuracy of the two sensor installation modes is not significant. After the decision tree is pruned according to the recognition results of the verification set, the recognition object set is recognized. The accuracy is shown in Tables 7 and 8.

After pruning, the recognition accuracy of the decision tree on the recognition object set is higher than that of the verification set. Among them, the average recognition accuracy of the placement of the lower limb and forearm on the same side is 96.49%, and the average recognition accuracy of the placement on the opposite side is 96.20%, which are higher than that of 93.85% and 94.64% before pruning. Then, compare the recognition accuracy of the two decision trees generated under the same side and different side placement. Through the data in Tables 8 and 9, it can be seen that the recognition accuracy of the same side of the forearm sensor and the lower leg sensor is slightly higher than that of the opposite side, but the difference is very small whether before or after pruning. Therefore, it can be considered that the accuracy of human body recognition under the two sensor placement methods is basically the same.

According to the performance of the above decision tree in the verification set and the recognition object data set, it can be concluded that for the decision tree classification, although the action has a certain asymmetry, the recognition accuracy of the sensor placed at the left and right lower legs is almost the same, and there is not much difference. It can be considered that the two sensor placement positions using decision tree algorithm have the same effect on action recognition. The reason is analyzed here: when the human body is standing, walking, and running, no matter whether it is dribbling or not, the motion symmetry of its left and right legs remains good, and there is no obvious difference in motion mode. Therefore, there is no significant difference in recognition efficiency between the sensor at the lower leg and the sensor at the forearm. Next, the training time and recognition time of each action of the decision tree are studied: the training time is timed from after reading the data into the memory, before starting the training, to the end after the pruning of the decision tree is completed.  Table 9 shows the comparison of training time under two sensor placement modes.

For two decision trees, each decision tree is trained with a total of 675 groups of data, and a total of 342 groups of data are verified and pruned. The two decision trees take 7.17 s and 7.32 s to complete the training process, respectively. It can be seen that when the number of training groups is equal, the training time of the two placement methods is close, so it can be considered that the two placement methods have little effect on the training speed of decision tree.

## 5. Conclusion

For innovation in the research process, an algorithm for identifying the characteristics of weightlessness state is proposed. Compared with the previous algorithm for estimating the take-off speed through the acceleration integral to identify the take-off height, this algorithm has lower complexity by identifying the “weightlessness characteristics.” Through experimental verification, it can achieve higher recognition accuracy. Through the subject analysis and research, this paper comes to the conclusion that the two sensor placement methods have the same recognition accuracy of the subject target action, and the recognition effect of SVM classifier is better than that of decision tree classification. It is of great research value to study the direction of movement recognition in human body. First of all, in addition to acceleration, speed data and angular data can be introduced into the work of recognition research. In addition, a variety of sensors, classifiers, and sensor combination methods can also be applied in the recognition research of human actions.

## Figures and Tables

**Figure 1:** A manufacturing method of physical training monitoring system.

**Figure 2:** Action recognition process.

**Figure 3:** Overall framework of the system.

**Figure 4:** Schematic diagram of coordinate system: (a) sensor motion coordinate system; (b) ground coordinate system.

**Table 1:** Sensor data calibration.

8.7348	0.0121	16.2010	0.0110	-10.5738	0.0108	-76.8471	0.1311
8.7351	0.0110	16.1732	0.0116	-10.5852	0.0101	-77.0150	0.1580
8.6560	0.0117	16.1753	0.0107	-10.5852	0.0105	-76.7703	0.1420
8.6541	0.0110	-3.2355	0.0053	-6.4005	0.0086	122.4826	0.1087
8.6502	0.0112	-3.3001	0.0048	-6.3853	0.0081	122.3672	0.1112
8.8780	0.0118	-123.1023	0.1100	-8.3701	0.0101	-31.4828	0.1238
8.8801	0.0125	-123.1687	0.1107	-8.3733	0.0110	-31.4766	0.1400
8.8766	0.0114	-123.1771	0.1062	-8.3721	0.0088	-31.4802	0.0260

**Table 2:** PC configuration required for experiment.

Configuration name	Specific model and performance
CPU	Intel Core i7-6700HQ main frequency 2.6 GHz, 4 cores, maximum frequency 3.1 GHz
Memory	ADATAXPG8GDDR42400MHz ×2, actual operating frequency 2133 MHz
System	Windows 10 professional x64
Experimental platform	MATLAB2017b (x64)

**Table 3:** Accuracy of weightlessness feature extraction and recognition.

Total number of groups	Correct quantity	Number of errors	Correct rate
150	148	2	98.67%

**Table 4:** Average time for weight loss feature recognition.

Total number of groups	Average time
150	0.03327 ms

**Table 5:** Recognition accuracy of ipsilateral placement of decision tree verification set.

Action	Other misoperation identification	Error	Error condition	Correct rate
Stand	0	0	Nothing	100%
Standing dribble	0	0	Nothing	100%
Free throw	1	0	Nothing	100%
Jump shot	1	2	Jump once, free throw twice	97.44%
Jump	1	1	Jump shot once	92.31%
Walk	1	2	Run twice	94.88%
Run	4	0	Nothing	90.48%
Walking dribble	1	3	Walk once and dribble twice	89.74%
Running dribble	2	3	Carry away once and run twice	87.5%

**Table 6:** Recognition accuracy of different side placement of decision tree verification set.

Action	Other misoperation identification	Error	Error condition	Correct rate
Stand	0	0	Nothing	100%
Standing dribble	0	0	Nothing	100%
Free throw	1	0	Nothing	97.44%
Jump shot	0	3	Jump twice and free throw once	92.11%
Jump	2	0	Nothing	95.00%
Walk	2	1	Run once	92.50%
Run	3	1	Walk once	92.68%
Walking dribble	1	2	Walk once and dribble twice	92.31%
Running dribble	1	3	Carry away once and run twice	89.74%

**Table 7:** Recognition accuracy of ipsilateral placement mode of object set identified by decision tree.

Action	Other misoperation identification	Error	Error condition	Correct rate
Stand	0	0	Nothing	100%
Standing dribble	0	0	Nothing	100%
Free throw	1	0	Nothing	97.37%
Jump shot	1	1	Free throw once	94.74%
Jump	0	1	Jump shot once	97.30%
Walk	1	0	Nothing	97.37%
Run	1	0	Nothing	97.37%
Walking dribble	1	2	Walk once and dribble once	92.11%
Running dribble	1	2	Transport once and run once	92.11%

**Table 8:** Recognition accuracy of different side placement methods of object set identified by decision tree.

Action	Other misoperation identification	Error	Error condition	Correct rate
Stand	0	0	Nothing	100%
Standing dribble	0	0	Nothing	100%
Free throw	1	0	Nothing	97.37%
Jump shot	1	2	Free throw once and jump once	92.11%
Jump	1	0	Jump shot once	97.37%
Walk	1	0	Nothing	97.37%
Run	1	1	Run once	94.74%
Walking dribble	1	1	Walk once	94.74%
Running dribble	1	2	Carry away once and run twice	92.11%

**Table 9:** Decision tree training schedule.

Decision tree	Corresponding placement mode	Total training time
*A*	Ipsilateral placement	7.16701 s
*B*	Different side placement mode	7.32387 s

## Data Availability

No data were used to support this study.
